# Region-Based Convolutional Neural Network-Based Spine Model Positioning of X-Ray Images

**DOI:** 10.1155/2022/7512445

**Published:** 2022-06-17

**Authors:** Le Zhang, Jiabao Zhang, Song Gao

**Affiliations:** ^1^Department of Radiology, Qingdao Municipal Hospital, Qingdao University, Qingdao, China; ^2^University College London, London, UK; ^3^Department of Obstetrics and Gynecology, Shengjing Hospital of China Medical University, Shenyang, China

## Abstract

**Background:**

Idiopathic scoliosis accounts for over 80% of all cases of scoliosis but has an unclear pathogenic mechanism. Many studies have introduced conventional image processing methods, but the results often fail to meet expectations. With the improvement and evolution of research in neural networks in the field of deep learning, many research efforts related to spinal reconstruction using the convolutional neural network (CNN) architecture of deep learning have shown promise.

**Purpose:**

To investigate the use of CNN for spine modeling.

**Methods:**

The primary technique used in this study involves Mask Region-based CNN (R-CNN) image segmentation and object detection methods as applied to spine model positioning of radiographs. The methods were evaluated based on common evaluation criteria for vertebral segmentation and object detection. Evaluations were performed using the loss function, mask loss function, classification loss function, target box loss function, average accuracy, and average recall.

**Results:**

Many bony structures were directly identified in one step, including the lumbar spine (L1-L5) and thoracic spine (T1-T12) in frontal and lateral radiographs, thereby achieving initial positioning of the statistical spine model to provide spine model positioning for future reconstruction and classification prediction. An average detection box accuracy of 97.4% and an average segmentation accuracy of 96.8% were achieved for the prediction efficacy of frontal images, with good image visualization. Moreover, the results for lateral images were satisfactory considering the evaluation parameters and image visualization.

**Conclusion:**

Mask R-CNN can be used for effective positioning in spine model studies for future reconstruction and classification prediction.

## 1. Introduction

Scoliosis is defined as a C- or S-shaped lateral spine curvature greater than 10°. Adolescent scoliosis is a common three-dimensional deformity of the spine that manifests as a disease with abnormal spinal sequences in the coronal, sagittal, and transverse planes. Scoliosis is classified as idiopathic, congenital, or neuromuscular, depending on its etiology.

Cases of scoliosis where the pathogenic mechanism is unclear are classified as idiopathic scoliosis, currently accounting for over 80% of cases. In the United States, the prevalence of adolescent idiopathic scoliosis is 1-3% [1]. Although the incidence of congenital scoliosis is much lower than that of idiopathic scoliosis, congenital scoliosis has a more significant impact on the physical and mental health of patients because it is accompanied by structural deformities such as vertebral hypoplasia [2]. Without timely intervention and treatment during spinal growth and development, the angle of scoliosis gradually worsens, leading to spine deformity, ribcage deformity, and possibly pain and even nerve compression in the shoulder, back, and thoracic and lumbar spine and respiratory distress [3, 4]. Given the high incidence and impact on the physical and mental health of adolescents, scoliosis has been listed as one of the four major diseases of adolescents and has received widespread attention from all segments of society. Therefore, the classification and prediction of the tendency of scoliosis through technology are of great interest.

Three-dimensional reconstruction of the spine is important for future scoliosis staging and outcome prediction. Further, the classification of scoliosis is an important foundation for determining an appropriate treatment plan. Currently, the classification of scoliosis and treatment guidelines are based on 2D spine radiographs. However, scoliosis manifests as a disease with abnormal spinal sequences in the coronal, sagittal, and transverse planes and the three-dimensional spatial structure of the abnormal vertebrae. Consequently, the diversity in curve types and morphology cannot be appreciated through 2D radiographs alone, possibly leading to misinterpretation of different scoliosis deformities with similar 2D parameters. Artificial intelligence technology can be used for objective measurement and analysis of the characteristic parameters of scoliosis and to achieve accurate classification based on the characteristic parameters. However, the progression and prognosis of scoliosis are difficult to determine even after accurate and objective scoliosis classification owing to vertebral growth disorders causing imbalances in spinal growth and other causes. Therefore, spine model positioning is important for subsequent studies requiring 3D reconstruction of the spine for scoliosis classification and treatment.

In this paper, we propose a training network model based on the Mask Region-based convolutional neural network (Mask R-CNN) architecture for one-step direct identification of spine models in human frontal and lateral X-ray images, including the lumbar spine (L1-L5) and thoracic spine (T1-T12). In addition, we provide the initial positioning of statistical spine models, thus providing spine model positioning for future reconstruction and classification prediction.  Figure 1 shows a flow diagram of this study.

## 2. Related Work

Many studies have introduced conventional image processing algorithms for spine model positioning, including using conventional segmentation algorithms such as the Canny edge detector, the active contour (snake) algorithm [5], and the generalized Hough transform for automatic segmentation of vertebral projections. Subsequently, in conjunction with a generic 3D model of the spine and segmented vertebral radiograph images, 3D/2D alignment is used to separately estimate the position of each vertebra. However, the results of these attempts have predominantly been inadequate. Difficulties such as low contrast in fluoroscopic images and overlapping or concealed tissue structure make conventional segmentation algorithms ineffective. In addition, applying 3D/2D alignment to each vertebra is time-consuming, and the local alignment results are incompatible with the overall structure of the spine.

With the continued improvement and evolution of research in neural networks, encouraging research results have been obtained in academic studies. Many research studies related to spinal reconstruction have used the CNN architecture. Arif et al. employed a CNN-based segmentation model to segment the spine in lateral radiographs and obtained ideal experimental results with high accuracy [6]. However, because of the single output of the CNN, the boundaries of overlapping parts are difficult to determine. The individual optimization of CNNs in multiple fragmented processes increases algorithm complexity and makes quality control difficult. In contrast, the primary technique used in our study is Mask R-CNN-based image segmentation and object detection methods as applied to spine model positioning in X-ray images.

### 2.1. Developments in 3D Spine Reconstruction

The evolution of 3D spine reconstruction algorithms has been following the technical route of gradually increasing the fine-tuning parameters of 3D spine models while reducing manually controllable parameters during the reconstruction process. Commonly used spine models are typically obtained by generating 3D models from boundaries outlined in sectioned computed tomography or magnetic resonance imaging images [7]. Owing to differences in algorithms and use cases, the generated 3D models are of three primary types: point cloud, mesh, and nonuniform rational B-splines [7–10]. Earlier reconstruction algorithms required manually locating 0-30 bony marker points for each vertebra in projection images to predict its 3D coordinates and generate a 3D mesh model for morphological adjustments and eventually complete the reconstruction [11]. Various statistical models based on standard a priori databases have since emerged to reduce the processing time. Semiautomatic methods using these models require only a small number of parameter inputs to predict the geometric parameters of a 3D model of the spine. There are two types of models: parametric dimensionality reduction models and parametric spine models. The parametric dimensionality reduction model is a principal component analysis model or a multiple linear regression model aimed at reducing the parameter inputs [12, 13].

Early parametric spine models generally utilized six marker points per vertebra, which were sufficient to generate the entire point cloud model of the spine. However, such models lacked parametric degrees of freedom and could not fully represent a fine-grained 3D mesh model [12, 13]. To address this issue, Humbert et al. made modifications and proposed a more mature and easy-to-use semiautomatic reconstruction algorithm [14]. Their method accounts for both the longitudinal and transverse geometric morphologies of the spine. The longitudinal morphology is determined by a line through the center of the vertebral body, whereas the transverse morphology is determined according to a simplified parametric model of the local deformation of the vertebrae. This two-level parametric description is still used today. However, this semiautomatic method has different sensitivities to the location of individual marker points for manual input. Operator interaction with the iterative input process is often nonintuitive and time-consuming, at approximately 11.5 min on average [15].

Recently, Parent et al. proposed a CNN-based architecture for bony anatomical landmark detection in frontal and lateral images. These include the vertebral arch and the vertebral endplate, which allow for finer adjustments in the reconstructed model [16]. Aubert et al. conducted a study based on bony landmark detection and achieved rapid automated reconstruction within 2 minutes [17]. However, individual optimization of CNNs in multiple fragmented processes increases algorithm complexity and makes quality control difficult; in addition, such algorithms still suffer from low contrast caused by overlapping tissue structures.

### 2.2. Developments in Spine Model Positioning in Spinal Reconstruction

Before spinal reconstruction, the coordinate system and geometric scale relationships must be defined based on the accurate positioning of bony structures such as the femoral head, sacroiliac joint, and sacral endplate. In semiautomatic reconstruction methods, these data are manually marked. In a recent automatic reconstruction study, Aubert et al. used a multilevel, mutually independent CNN model to determine these bony structures separately to improve the accuracy of parameter estimates through multiple adjustments [17]. However, training multiple CNNs separately in this manner makes it difficult to achieve global cooperative training optimization and poses problems for quality control of the algorithm in clinical applications.

In recent years, the accuracy and speed of multitarget recognition frameworks in the field of computer vision have reached unprecedented levels owing to the development of deep learning [18]. In contrast to conventional CNN, the R-CNN architecture can classify multiple regions of interest in the input image based on a feature map obtained from the shared CNN training, eventually resulting in multitarget recognition and positioning. Mask R-CNN can further segment the object boundaries to facilitate higher-order in-depth analysis. Therefore, we aimed to use the R-CNN architecture to train the network model to directly identify many bony structures, including lumbar and thoracic vertebrae in frontal and lateral X-ray images in a single step, thereby achieving the initial positioning of the statistical spine model.

Thus, the present study differs from recent studies in that the Mask R-CNN architecture is used to train the network model to directly identify many bony structures, including the thoracic spine and lumbar spine, in frontal and lateral radiographs in a single step, while providing the initial positioning of the statistical spine model, thereby simplifying the positioning process.

## 3. Materials and Methods

### 3.1. Preprocessing and Serial R-CNN Models

#### 3.1.1. Preprocessing

In this study, we preprocessed the human X-ray images acquired before putting the dataset into a standard format. The X-ray images used were anonymized X-ray images in DCM format. First, ImageJ was used to convert the X-ray images from DCM to JPG format.

#### 3.1.2. R-CNN

R-CNN uses an object recognition method on regions based on sliding windows. First, category-independent sets of candidate regions are generated on a given image, and each candidate region set is labeled with a category and a bounding box. Next, for each candidate region, a CNN is used to extract a fixed-length eigenvector. A support vector machine (SVM) classifier is trained for each category to determine the probability that the eigenvectors belong to each category. The eigenvectors output from the CNN are fed into the SVM classifier to predict the probability that the objects in the candidate regions belong to each category.  Figure 2 depicts the R-CNN model.

#### 3.1.3. Faster R-CNN

Faster R-CNN improves upon R-CNN by adding a region proposal network (RPN) for detecting target regions instead of using selective search to extract candidate regions. The RPN is a fully convolutional network that can exclude meaningless regions not belonging to any target category, reduce the number of proposed regions generated, and increase the speed of candidate region generation while ensuring precise object detection.  Figure 3 illustrates the Faster R-CNN model.

#### 3.1.4. Mask R-CNN

Mask R-CNN adds a feature pyramid network (FPN) to overcome the limitations of region transformation, improve algorithm efficiency, and effectively use the pixel-level location information of the training data image labels. Introducing a residual network as deep semantic information prevents the vanishing gradient problem, thereby improving model accuracy.  Figure 4 illustrates the Mask R-CNN model algorithm.

Mask R-CNN uses a residual network to better utilize the features extracted from deep convolution. The RoIPool is replaced with a region of interest alignment layer using a bilinear difference method instead of roughly selecting a value to substitute for the value of the entire region because each region also has a size gap. The bilinear interpolation method is extended by calculating the linear difference in each of the two directions and is more appropriate for mapping the region of interest to the feature map by performing bilinear interpolation for each point. The output of the region of interest alignment layer contains the same shape as the feature map and can be used for mask classification prediction and the bounding-box shape of the region of interest in all regions of interest. In addition, the pixel-level mask position of the target can be predicted using the full CNN. Improving the RPN to FPN connects different convolutional layers to better identify features at different scales.

### 3.2. Basic Principles of the Mask R-CNN Model

#### 3.2.1. Spine Positioning Model Design

As shown in Figure 5, the spine X-ray image positioning network structurally contains modules such as a CNN backbone, feature map processing, mask calculation, bounding-box prediction, and category prediction. First, spine radiographs are input into the Mask R-CNN, and then, the convolutional layer of the CNN backbone extracts features from the input image. Next, the candidate regions of the vertebrae are extracted using the RPN, with feature maps of different scales generated by the FPN. Finally, the feature map set is passed into the head of the network, comprising three branches: mask branch that calculates the 2D mask of vertebra instances in each region of interest, box regression branch to determine the extent of the vertebra box, and classification prediction branch, for instance, classification prediction.

#### 3.2.2. Convolutional Computation

At the base of the model is a convolutional backbone that extracts the input image feature map through layer-by-layer convolutional computation. The entire spine model localization process must undergo convolutional computation before subsequent classification, vertebral mask generation, and vertebral box computation can be performed. Convolutional computation often requires improvement. Simply increasing the network depth results in the vanishing gradient problem, causing the accuracy of results to gradually tend toward fitting after increasing to some value, and the accuracy will instead keep decreasing as the network depth increases.

In deep convolutional networks, although the number of convolutional layers and the feature expression capability increase with increased convolutional computation, the vanishing gradient problem often remains. The deeper the layers of an ordinary neural network, the closer the initialization parameters are to zero. As the training of neural networks usually involves a backpropagation algorithm for chain product derivation, the more the gradient of the shallow layer tends to zero as the information is propagated forward when the parameters of the shallow layer are updated, the more the gradient eventually disappears. In other words, the accuracy tends to fit after the depth of the model increases to a certain limit, and the accuracy decreases if the convolution depth of the network continues to increase. Therefore, the Mask R-CNN model introduces a residual convolutional network (ResNet) to effectively avoid the vanishing gradient problem and improve model accuracy [19–21]. Equation (1) is the mathematical representation of the residual module. The input data *x*_*i*_ of the residual block are identity mapped to *w*_*i*_*x*_*i*_ (*W* = 1 without dimensional conversion) through a shortcut connection, and *x*_*i*_ is convolved and activated by the activation function *G*_*i*_ to output the residual value *F*(*x*_*i*_, *G*_*i*_).

(1) $$\begin{array}{c} x_{i+1}=F\left(x_{i},G_{i}\right)+Wx_{i}. \end{array}$$

Here, *x*_*i*_ is the data input of the residual block at layer *i*, *G*_*i*_ is the activation function, *F*(*x*_*i*_, *G*_*i*_) is the residual value, *W* is the constant mapping parameter (usually 1), and *x*_*i*+1_ is the input of the residual block at layer *ⅈ* + 1.

Any layer *x*_*k*_ deeper than layer *x*_*i*_ can be represented as *x*_*i*_ (Equation (2)). The gradient *dl*/*dx*_*i*_ of the loss function for *x*_*i*_ is found using Equation (3) with *W* as one.

(2) $$\begin{array}{c} x_{k}=\overset{k-1}{\underset{j=i}{\sum }}F\left(x_{i},G_{i}\right)+x_{i}, \end{array}$$

(3) $$\begin{array}{c} \frac{\text{ⅆ}l}{\text{ⅆ}x_{i}}=\frac{\text{ⅆ}l}{\text{ⅆ}x_{k}}\frac{\text{ⅆ}x_{k}}{\text{ⅆ}{\text{x}}_{\text{i}}}. \end{array}$$

Here, *x*_*k*_ is the residual block input value of layer *k*(*k* > *i*), *x*_*j*_ is the residual value from layer *j* to layer *j* − 1, *G*_*j*_ is the activation function from layer *i* to layer *k* − 1, and *F*(*x*_*i*_, *G*_*i*_) is the residual value from layer *i* to layer *k* − 1.

Equation (2) is substituted into Equation (3) to obtain Equation (4). Equation (4) shows that the gradient of the deeper layer *x*_*k*_ can be transferred to any layer *x*_*i*_ that is shallower than *x*_*k*_. In addition, as the constant one in the parentheses and the product calculation in the conduction become a summation, its gradient never disappears regardless of the depth of the network layers.

(4) $$\begin{array}{c} \frac{\text{ⅆ}l}{\text{ⅆ}x_{i}}=\frac{\text{ⅆ}l}{\text{ⅆ}x_{k}}\frac{\text{ⅆ}\left(\sum_{j=i}^{k-1}F\left(x_{i},G_{i}\right)+x_{i}\right)}{\text{ⅆ}x_{i}}=\frac{\text{ⅆ}l}{\text{ⅆ}x_{k}}\left(1+\frac{\text{ⅆ}\sum_{j=i}^{k-1}F\left(x_{i},G_{i}\right)}{\text{ⅆ}x_{i}}\right). \end{array}$$

#### 3.2.3. Multiscale Processing

Usually, image targets have different scale sizes at the time of acquisition, and the objects in the dataset have different scales and sizes. A general dataset does not capture all image attributes, with objects of sizes smaller than the step size of the convolutional network not recognized effectively because they are ignored; this phenomenon is known as the multiscale problem. Vertebrae exist in different sizes, thus causing multiscale problems in training and recognition scenarios. FPNs using Fast R-CNN can effectively solve the multiscale problem [22–24]. As shown in Figure 6, FPNs employ a double pyramidal structure where they use lateral connections and top-down paths together through a simple merging layer, which is highly effective for feature processing.

The left pyramid is a conventional feature map CNN, and the feature map shrinks layer by layer with the number of convolutions. The classification task cannot be completed because the initial semantic information and features obtained from the bottom feature map after convolutional computation feature extraction in the initial convolutional layer are not sufficiently strong. The deep feature map has stronger semantic information and features; FPN exploits this key feature to capture stronger semantic information from the deep feature map and use it for the classification task through the path connections of the pyramid. However, the middle pyramid reverse samples the convolved image from top to bottom and enhances the expression of spatial and semantic information at different scales for each layer on the right side of the pyramid to detect small-scale targets by scaling up the feature map and then summing the elements with each pixel point of the feature map on the left side of the next layer without increasing the number of operations. The FPN takes the feature maps of images to the deepest layer of the network through a top-down connection path.

The FPN architecture cleverly combines lateral and top-down connectivity paths, allowing the extraction of deeper feature semantic information from images, feature fusion, and multiscale feature output, preventing the loss of semantic information caused by the limitations of existing processing. In scenarios where vertebral bone recognition is performed, the FPN model can exploit its multiscale recognition and increase the probability of detecting small-scale vertebral bone objects in images.

#### 3.2.4. Loss Calculations

After feature region extraction and screening, the network head separately calculates the mask, box, and classification loss values for the feature regions. The classification loss value is the logarithmic loss that divides the object and nonobject classes after binary discrimination of the target. The segmentation error is the loss calculated for each class of the mask. The innovation of the segmentation error is that if the region of interest is detected to belong to a certain category, the relative entropy error of that category is used for the calculation. Kaiming et al. empirically demonstrated that selecting the sum of the classification, box, and mask loss values (Equation (5)) as the overall loss value in model training yields good results for multiple datasets [25].

(5) $$\begin{array}{c} L=L_{\text{cls}}+L_{\text{box}}+L_{\text{mask}}. \end{array}$$

Here, *L*_cls_ is the loss value calculated using classification, *L*_box_ is the loss value calculated using the bounding-box, *L*_mask_ is the loss value calculated using the mask, and *L* is the overall loss value of the network.

## 4. Results and Discussion

### 4.1. Experimental Environment

#### 4.1.1. Database Construction

The human spine images acquired for the experiments were anonymized and divided into frontal and lateral views. One category comprised human X-ray images converted from DCM to JPG format using ImageJ; these images were used to study the images to be processed. The other category comprised ground-truth images obtained by converting DCM to JPG format using ImageJ, adding mask annotation using LabelMe image annotation software with alignment using ImageJ, and generating mask images and mask annotated images required for model training. The images of the 12 thoracic vertebrae and the 5 lumbar vertebrae were labeled, with different vertebrae being labeled with different colors. Labeling was performed based on vertebra identification according to human anatomical morphology, starting from T1 and labeling the thoracic vertebrae (T1-T12) and the lumbar vertebrae (L1-L5).

#### 4.1.2. Data Settings and Augmentation

In this study, there were 250 frontal and lateral X-ray images of the human spine. In order to obtain standard X-ray images, we took the following measures. First, we minimized the overlap between the bone and soft tissue of the shoulder joints and the upper thoracic spine by standardizing the position and method of radiography. Second, we carefully observed each image and reject images with artifacts. Finally, we adjusted the contrast of the images to obtain the best experimental results.

ImageJ was used for grayscale adjustment to facilitate annotation. The data were created in the COCO dataset format, and the dataset was divided into 170 images for the training set in the frontal and lateral position, 6 images for the validation set in the frontal position, 5 images for the validation set in the lateral position, and 70 images for the test set.

#### 4.1.3. Data Settings and Augmentation Experimental Platform Construction and Environment Configuration

Python programming language and Linux operating system were used in this study. The environment was configured to use Python, PyTorch, and CUDA to build the Mask R-CNN models using a ResNet-50 convolutional backbone. Two GPUs were used for training.

### 4.2. Analysis of Experimental Results

#### 4.2.1. Frontal Spine Radiograph Experiments

In this study, we first trained and tested frontal spine radiographs, and the model was trained with the Mask R-CNN on the existing training set.  Figure 7 shows the changes in loss values.

The experimental results show that the loss function, mask loss function, regression loss function, and classification loss function converge after approximately 10,000 iterations of training on frontal radiographs. After model training, frontal spine radiographs were tested, the test set was selected, and the results were obtained, as shown in Figures 8 and 9. For spine model positioning, the vertebrae were identified during object detection, with semantic and instance segmentation of the vertebrae also achieved at the thoracic and lumbar levels. As shown in Figure 8, the thoracic vertebrae (T1-T12) and the lumbar vertebrae (L1-L5) were individually segmented in the semantic segmentation, and the detection box was distinguished between the thoracic vertebrae and lumbar vertebrae. In the instance segmentation in Figure 9, the vertebrae are segmented into different colors, and the detection box distinguishes between the thoracic vertebrae and lumbar vertebrae.

Table 1 shows the values of the average recall (AR, the average value at a threshold of 0.5-0.95 as the IoU), the average precision (AP) 50 (at an IoU of 0.50), and accuracy for the segmentation and object detection box using the ResNet-50 CNN. The table indicates good test results with the frontal radiographs, with the accuracy of both vertebral segmentation and vertebral object detection boxes reaching 99.8%. The average accuracy of vertebral segmentation was 96.8%, and the AR was 62.2%. The average accuracy of the object detection box was 97.4%, and the AR was 70.5%. As the vertebrae in the frontal human spine radiographs are relatively clearly visible and virtually completely unobstructed by tissue or bone, it had good performance in both the labeling and training tests.

Spine model positioning of frontal spine radiographs based on the Mask R-CNN architecture provides good performance for recognition of vertebrae, including detection of frontal spine radiographs by segmentation and the object detection box.

#### 4.2.2. Lateral Spine Radiograph Experiments

In this study, lateral spine radiographs continued to be used as test objects. While labeling the lateral spine radiographs, we found that some of the vertebral structures were almost invisible because they were obscured by the body, especially in the upper thoracic vertebrae, where the vertebral column was nearly invisible during labeling and could only be judged by the scale bar. This made it difficult to label, train, and make predictions using lateral radiographs, thus increasing the difficulty of the experiment.

The model was trained with the Mask R-CNN on the existing training set of lateral radiographs.  Figure 10 shows the changes in loss values.

After 24000 iterations of model training, the test set of lateral spine slices was tested; the results obtained are shown in Figures 11 and 12. The test results of spine model positioning based on the Mask R-CNN architecture, including detection of lateral spine radiographs by segmentation and the object detection box, were unsatisfactory. Although the vertebrae can be identified in object detection and semantic and instance segmentation of the thoracic and lumbar vertebrae was performed, there were cases of incomplete image segmentation. In addition, although the object prediction box predicted the vertebra position correctly, the classification of thoracic and lumbar vertebrae was incorrectly predicted.

Table 2 shows the values of the AR (the average value at a threshold of 0.5-0.95 as the IoU), the AP75 (at an IoU of 0.75), and accuracy for the segmentation and object detection box using the ResNet-50 CNN. The table indicates satisfactory test result parameters with the lateral radiographs, with an average accuracy of vertebral segmentation of 81.6% and an AR of 63.8%. The average accuracy of the object detection box was 90.1%, and the AR was 90.0%.

The experimental results of spinal model positioning of lateral images are analyzed as follows:

1. In clinical work, because the first to third thoracic vertebrae overlap with the shoulder joints on both sides in the lateral radiographs, sometimes, part of the thoracic vertebrae cannot be clearly displayed. In this case, it is difficult for even experienced radiologists to accurately label this part of the thoracic vertebrae on the lateral radiographs. Consequently, there were difficulties in labeling, training, and prediction in the experiments. The loss was still approximately 0.08 after training for 24000 iterations, and the rate of decline was also slow. This made the final prediction results not reach the best state, resulting in inaccurate segmentation and classification reversal errors
2. In this study, the training of lateral images required twice as many iterations as frontal images to achieve a similar loss. The loss function was not yet optimal, and the existing experimental results could not yield completely correct results for the positioning of the lateral image spine model. The prediction results have some incomplete skeletal segmentation, and the reason for the reversed thoracic and lumbar classification prediction warrants further investigation. To solve the problems, more training or comparison iterations or a more efficient training backbone network may be required
3. The dataset partitioning performed in this study still needs to be improved as the excessive number of training sets without a reasonable proportion of datasets may lead to errors in the evaluation parameters. In future studies, a more reasonable dataset division for training, testing, and validation should be performed. In addition, constructing a larger database will also help improve the accuracy of experimental results

## 5. Conclusions

In this study, we performed human X-ray image spine model positioning based on an R-CNN. We focused on object detection and image segmentation and the effect of Mask R-CNN on human radiograph spine model positioning, detection, and segmentation. Considering application directions, we focused on radiographic spine model positioning.

Python language was used to configure Mask R-CNN, including FPN with ResNet-50 and other network architectures, to conduct extensive training on a large amount of data from frontal and lateral slices and testing on spine radiographs. The segmentation and detection results of many bony structures, including L1-L5 in the lumbar spine and T1-T12 in the thoracic spine, were obtained in a single step. Considering the experimental results, the prediction efficacy for frontal images and image visualization was good, with an average detection box accuracy of 97.4% and an average segmentation accuracy of 96.8%. The results for lateral images were satisfactory considering the evaluation parameters and image visualization, but the problem of classification and prediction errors warrants further attention. Overall, the study provides a basis for spine reconstruction, scoliosis classification, and scoliosis prediction and adds value to the research on automatic spine model positioning.

Based on the characteristics of the vertebrae in lateral radiographs of the spine, there are still many shortcomings in this study that must be addressed. In this study, the lateral images were often not as easily observed because the body blocked the thoracic spine, leading to inaccurate labeling, which affected training and testing. We reduced errors by standardizing the photographic position, adjusting the contrast of the images, and using the scale bar. There were still shortcomings in the positioning and segmentation of the lateral images in this study. In the future, more network architectures such as ResNet-101 and VGG neural networks should be used as convolutional backbones for comparison, with the network parameters adjusted more carefully to select the optimal network architecture to solve the problems of incorrect classification and segmentation of lateral radiographs.

## Figures and Tables

**Figure 1:** Flow diagram of our Mask R-CNN-based spine model positioning study.

**Figure 2:** Schematic of R-CNN model.

**Figure 3:** Schematic of the Faster R-CNN model.

**Figure 4:** Schematic of the Mask R-CNN model.

**Figure 5:** Schematic of spine model positioning network.

**Figure 6:** Schematic of the feature pyramid network (FPN).

**Figure 7:** Change in loss values for frontal image training set.

**Figure 8:** Example of test results of frontal image semantic segmentation.

**Figure 9:** Example of test results of frontal image instance segmentation.

**Figure 10:** Change in loss values for lateral image training set.

**Figure 11:** Example of test results of lateral image semantic segmentation.

**Figure 12:** Example of test results of lateral image instance segmentation.

**Table 1:** Parameters for evaluating the experimental results of the spine model positioning (frontal images).

	Accuracy	IoU = 0.5 Average precision (AP50)	Average recall (AR)
Spine segmentation	99.8%	96.8%	62.2%
Detection box	99.8%	97.4%	70.5%

Note: average recall (AR) represents the average IoU in the range of 0.5-0.95 at intervals of 0.05.

**Table 2:** Parameters for evaluating the experimental results of spine model positioning (lateral images).

	Accuracy	IoU = 0.75 Average precision (AP75)	Average recall (AR)
Spine segmentation	99.8%	81.6%	63.8%
Bounding box	99.8%	90.1%	90.0%

Note: average recall (AR) represents the average IoU in the range of 0.5-0.95 at intervals of 0.05.

## Data Availability

The data used to support the findings of this study are available from the corresponding author upon request.
